# Applied Research on the Combination of Weighted Network and Supervised Learning in Acupoints Compatibility

**DOI:** 10.1155/2021/4699420

**Published:** 2021-10-29

**Authors:** Xia Qiu, Xiaoying Zhong, Honglai Zhang

**Affiliations:** College of Medical Information Engineering, Guangzhou University of Chinese Medicine, Guangzhou 510006, China

## Abstract

To enhance the depth of excavation and promote the intelligence of acupoint compatibility, a method of constructing weighted network, which combines the attributes of acupoints and supervised learning, is proposed for link prediction. Medical cases of cervical spondylosis with acupuncture treatment are standardized, and a weighted network is constructed according to acupoint attributes. Multiple similarity features are extracted from the network and input into a supervised learning model for prediction. And, the performance of the algorithm is evaluated through evaluation indicators. The experiment finally screened 67 eligible medical cases, and the network model involved 141 acupoint nodes with 1048 edge. Except for the Preferential Attachment similarity index and the Decision Tree model, all other similarity indexes performed well in the model, among which the combination of PI index and Multilayer Perception model had the best prediction effect with an AUC value of 0.9351, confirming the feasibility of weighted networks combined with supervised learning for link prediction, also as a strong support for clinical point selection.

## 1. Introduction

Acupoint compatibility is the application of two or more acupoints under the principle of selecting acupoints, through which the synergy between the acupoints is strengthened and medical efficacy is achieved [1]. Acupuncture prescription, which has high clinical value, is the combination of clinical practice and TCM theories, including principle, method, prescription, and acupoint. Among them, the compatibility of acupoints is the basic element of acupuncture prescription, so most studies use acupuncture prescriptions as the basis for exploring the laws of acupoint compatibility. Acupoint compatibility is not a simple “1 + 1” in a mathematical equation, the number of acupoints is not directly proportional to the quality of the combination, and there are various methods of acupoint compatibility, such as distant and near acupuncture points, following the meridian and identifying the evidence, which makes the factors affecting the efficacy of acupoint compatibility unclear. How to effectively analyse the pattern of acupoint compatibility to enhance clinical efficacy has made acupoint compatibility a hot research topic.

The selection of acupoints for clinical treatment is mainly dependent on medical records and the clinical experience of the practitioner and is subjective and limited. With the development of information technology, the research of acupoint compatibility has made progress with the help of data mining technology, especially complex network technology that expresses the nonlinear and complex relationships between nodes by constructing network models. Zhen et al. [2] used quantitative indicators such as network topology and structural parameters to objectify and assess the collocation relationships between acupoints. Wen et al. [3] used the angle and direction of needling to construct a network model to explore the characteristics of moxibustion. Jiang et al. [4] constructed an acupuncture point network model and showed that the distal and proximal point allocation method is often applied in acupoints compatibility for hiccups. In reality, the acupoint network is not a single network: it is a reflection of the theory of TCM diagnosis and treatment, and most studies combining acupoint compatibility with complex networks have limitations such as a single model of the acupoint network, the degree of connection between acupoints is not quantified, and only the frequency of cooccurrence is used to show the pattern of acupoint coordination.

Link prediction is one of the cores of complex network research and can reveal the implicit connection rules of nodes in the graph. The research ideas and methods are derived from Markov chains and machine learning. Nowadays, it is widely used in many fields of research, such as disease networks [5], drugs networks [6], and social networks [7]. With the rapid development of machine learning, a large number of researches on the combination of supervised learning and link prediction have been conducted [6, 8–11]. Although link prediction has not been seen applied to acupuncture point networks in studies combining acupoint compatibility with complex networks, link prediction can effectively transform the problem of measuring the degree of relationship between nodes in a network into a problem of the likelihood of establishing links between nodes, which provides a new perspective on acupoint compatibility. To solve the problems above, this research is designed to construct a weighted complex network in order to abstract the actual acupuncture prescriptions for cervical spondylosis with the consideration of acupoints attributes. Based on weight, multiple types of features are extracted. In order to improve the depth of mining and explore the law of acupoint compatibility, the features are input into the supervised learning model for training and prediction, and the effects of features and models on forecasting performance are compared. The research is the preliminary exploration of intelligent acupoint selection and compatibility in TCM.

## 2. Weighted Network

### 2.1. Data Collection and Processing

From the platform of modern medical records cloud (http://www.yiankb.com/), the prescriptions of acupuncture and moxibustion used in cervical spondylosis were collected. To ensure the effectiveness of the network construction, it is necessary to collect the medical records of the patients who are diagnosed with cervical spondylosis. In the selection, the prescription should be clear, the treatment should be conducted mainly by acupuncture, and the condition of patient should be improved obviously. Finally, 67 medical records were collected, involving 115 acupoints and 1048 groups of acupoint combinations. The names of the acupoints were represented by the international code, and the extra points without international code were represented by Chinese Pinyin. Through *Python*, the medical records were revised with standardized names.

### 2.2. Network Construction

In the study, the acupoints extracted from the prescriptions of acupuncture treatment for cervical spondylosis were used to construct a weighted acupoint network. The weighted acupoint network was expressed as *G*=(*V*, *E*, *W*), where *V*, *E*, and *W* were the set of nodes in the network, the set of edge relations, and the set of weights, respectively. The process of constructing a weighted acupoint network model could be mainly divided into three steps. (1) Extract all the acupoints in the prescription to form a set of nodes (*V*). (2) Each two acupoints in a prescription were connected as an edge to form the edge subset. And as such, the total set of the relations was built (*E*). (3) The similarity between all acupoint nodes was calculated and was used as the weight to build the weight set (*W*). Finally, *V*, *E*, *W* were combined to construct a weighted network. As shown in Figure 1, the network was visualized through Gephi.

The weight was determined by the similarity between the acupoints. Based on the attributes of nodes, the similarity was shown in a numerical form. It is believed that [12] the meridians, body surface location, and deep structure of acupoints are the inherent attributes, and the indication is the functional attributes. And the understanding of the attributes could improve the syndrome differentiation and acupoint compatibility in clinical acupuncture and moxibustion treatment. In the research, the attributes of meridian, location, and indication were used to calculate the similarity. Refering to the textbook Acupuncture and Moxibustion, the attributes of acupoints in the prescription for the treatment of cervical spondylosis were summarized, including 15 types of meridians (14 meridians and extra acupoints), 63 locations, and 670 indications, as shown in Table 1. Combining the acupoints in the prescription for the treatment of cervical spondylosis, the vectorized acupoint attributes were calculated by the cosine similarity. And then, the similarity of the acupoint group was obtained. The calculation formula is shown in


(1) $$\begin{array}{c} \cos\left(x,y\right)=\frac{x\cdot y}{\left\|x\right\|\cdot \left\|y\right\|}. \end{array}$$

## 3. Link Prediction

Link prediction was mainly divided into four types of methods, including node attributes, network topology, machine learning, and maximum likelihood. Comparing to the difficulty of obtaining the information of node attributes, the method of link prediction, which is based on the network topology, can judge the possibility of establishing a connection between nodes clearly through the network structure [13]. Based on network topology, link prediction could also be divided into three research directions: local information, random walk, and path. In the link prediction of acupoint network, some features in the local information were selected. Although the link prediction was not based on node attributes, the essential information of attributes was not discarded. Instead, the information was converted into network weights, which was combined with network structure and machine learning in link prediction. In the weighted acupoint network that was constructed in the study, *E* was the set of all possible relationships between nodes, *E*_*y*_ was used to indicate that there existed edge in the network, and *E*_*n*_ was used to indicate that there did not exist edge in the network. The relationships of them were as follows: *E*_*y*_ ∪ *E*_*n*_=*E*， *E*_*y*_∩*E*_*n*_=∅. *E*_*y*_ was marked as a true positive sample, denoted by *y*=1, and *E*_*n*_ was marked as a false negative sample, denoted by *y*=0. And then, the compatibility of acupoints in clinical acupoint selection was transformed. Link prediction in the network was transformed into a second kind problem in machine learning.

### 3.1. Similarity Index

Local similarity is widely used in link prediction studies for its simplicity, scalability, and competitive prediction accuracy. The link prediction algorithm based on local similarity indexes predicts the likelihood of future links between *x* and *y* by the degree of intersection of the common neighbors of network nodes *x* and *y*. Common Neighbor (CN), Adamic-Adar (AA), and Resource Allocation (RA) are three common neighbor-based similarity indexes and Preferential Attachment (PA) is a preference connection similarity index. In this paper, four weighted similarity indexes were extracted from the weighted acupoint network structure and the fused four weighted similarity indexes were defined as PI, PI = {WCN, WAA, WRA, WPA}.

### 3.2. Local Similarity

#### 3.2.1. Weighted CN Index (WCN) [14]

(2) $$\begin{array}{c} s_{xy}=\sum_{z\in \in \Gamma \left(x\right)\cap \Gamma \left(y\right)}\frac{w_{xz}+w_{zy}}{2}, \end{array}$$

where Γ(*x*) and Γ(*y*) indicated the set of neighbor nodes of *x* and *y* and *w*_*xz*_ indicated the weight between nodes of *x* and *z*; when all the weight values were 1, formula (2) was equivalent to the unweighted CN index.

#### 3.2.2. Weighted AA Indicator (WAA) [14]

(3) $$\begin{array}{c} s_{xy}=\sum_{z\in \;\Gamma \left(x\right)\cap \Gamma \left(y\right)}\frac{w_{xz}+w_{zy}}{2\;\log\left(1+s_{z}\right)}, \end{array}$$

where *s*_*z*_ was the strength of node *z*. The degree of common neighbor nodes was considered by WAA. The contribution of the common neighbor with low degree was greater than the common neighbor with high degree. For example, compared to the users who listened to popular songs, the users who listened to niche songs were more likely to establish connections in a music recommendation system.

#### 3.2.3. Weighted RA Indicator (WRA) [15]

(4) $$\begin{array}{c} s_{xy}=\sum_{z\in \Gamma \left(x\right)\cap \Gamma \left(y\right)}\frac{w_{xz}+w_{zy}}{2s_{z}}. \end{array}$$

Nodes that were not directly connected in the network could transfer resources through common neighbors. In the process of transferring, the resources were allocated to neighbors equally according to the number of node neighbors. WRA was the number of resources finally received by the node.

### 3.3. Preference Connection Similarity

The weighted PA index (WPA) [16] indicated that the probability of establishing a connection between nodes was proportional to the product of the strength. And, the calculation formula is shown in

(5) $$\begin{array}{c} s_{xy}=\sum_{i\in \Gamma \left(x\right)}w_{ix}+\sum_{j\in \Gamma \left(y\right)}w_{jy}=s_{x}s_{y}. \end{array}$$

### 3.4. Evaluation Index

Area under ROC Curve (AUC), precision, and ranking score (recall) were the three evaluation indicators that were often used to measure the accuracy of link prediction algorithms. In the research, multiple supervised learning models were combined to make link prediction. So that model was one of the main influencing factors of the results. Therefore, three types of evaluation indicators, including AUC, recall, and F1-score, were used in the article to make a comprehensive evaluation of the results.

#### 3.4.1. AUC

In link prediction, an edge was randomly selected each time from the test set and the nonexistent edge set, and the fractional values of the two edges were compared. If the fractional value of edges in the test set is larger than that in the nonexistent edge set, 1 point will be added. If the fractional values are equal, 0.5 point will be added. The calculation formula is shown in formula (6), where *n* represented the number of independent comparisons, *n*′ represented the number of times that the fractional value of edges in the test set was larger than that in nonexistent edge set, and *n*^″^ represented the number of times that the fractional values of the two sets were equal.

(6) $$\begin{array}{c} \text{AUC}=\frac{n^{\prime }+0.5n^{\prime \prime }}{n}. \end{array}$$

#### 3.4.2. Recall

Recall indicated the number of cases that True Positive (TP) samples were predicted to be TP. There existed the following two situations: TP samples were predicted to be TP, and TP samples were predicted to be False Negative (FN). The calculation formula is shown as

(7) $$\begin{array}{c} \text{recall}=\frac{TP}{TP+FN}. \end{array}$$

#### 3.4.3. F1-Score

F1-score was the harmonic average of precision and recall. The calculation formula is shown in formula (8). P represented precision and *R* represented recall. When *α*=1, the formula was used for the calculation of F1-score.

(8) $$\begin{array}{c} F=\frac{\left(\alpha^{2}+1\right)P*R}{\alpha^{2}\left(P+R\right)}. \end{array}$$

### 3.5. Supervised Learning

The main differences between supervised learning and unsupervised learning existed in data labels. Supervised learning, which is mainly used to solve regression and classification problems, predicts unknown data with labeled data sets. The supervised learning algorithms that are commonly used are as follows: Support Vector Machine (SVM), Logistic Regression (LR), Multilayer Perception (MLP), k-Nearest Neighbor (KNN), Decision Tree (DT), and Adaptive Boosting (AdaBoost). Ying et al. [17] constructed three weighted disease networks derived from different medical data sets. The similarities were input as features into multiple supervised learning models to predict relationships of potential comorbidity. It was shown that the combination of global similarity features and supervised learning models could effectively improve the performance of the prediction algorithm. Zhao Sufen et al. [18] compared the application of 8 supervised learning algorithms on academic networks. The results showed that the performance of MLP was the best, and the performance of naive Bayes algorithm was the worst. The method of KNN was only better than naive Bayes. And the performance of other algorithms was almost the same. Considering the existed researches, four common algorithms were used in the study, including MLP, SVM, DT, and AdaBoost for link prediction of weighted acupoint networks. The steps of link prediction based on similarity features were divided into the following three steps.

The first step was data standardization. The similarity indexes extracted from the network were converted into a feature matrix. Due to the different dimensions of the matrix data, the matrix was standardized by Min-Max, and the data were linearly transformed. The data value was normalized from 0 to 1 to eliminate the impact of imbalance in proportion.

The second step was data balance. In the distribution of data categories, the ratio of TP to FN in the data set was 12 : 1. And there existed a typical data imbalance problem, which would cause the model prediction to be biased towards the side with a large sample size and would reduce the generalization ability of the model. So that the method of undersampling was adopted in the FN to achieve data balance in order to obtain 1 : 1 ratio of TP to FN.

The third step was model training. The data set was divided into training set and test set. Four supervised learning models were input in the training set for training. Finally, the test set was input to verify the results.

## 4. Results and Analysis

### 4.1. Experimental Setup

Based on the Jupyter notebook platform, Pandas and NumPy were used in the experiment to preprocess the data, NetworkX was used to build a weighted acupoint network. Four single similarity indexes and one fusion index were chosen as feature input to the supervised learning model, and the four models, MLP, SVM, DT, and AdaBoost, called by the scikit-learn (sklearn) package, were used to predict the similarity indexes and models in a two-by-two combination. RBF kernel function was selected and used in SVM model, and the parameters in the rest of the models were all default settings. The three evaluation indexes, AUC, recall, and F1-score, were chosen to evaluate the performance of the link prediction algorithm. In order to improve the accuracy of the results, ten-fold cross-validation was used to divide the data set, and the average value of ten times output was selected as the final result. And the three evaluation indicators were compared to evaluate the performance of the link prediction algorithm. The overall flow chart of the experiment is shown in Figure 2.

### 4.2. Experimental Results

The similarity indices were applied on the weighted acupoint network to evaluate the performance of various algorithms. The results are shown in Figures 3–5. AUC value was the standard for evaluating the predictive ability of the model. As shown in Figure 3, based on the similarity index, the AUC values predicted by each model were in the range from 0.5 to 1. The prediction accuracy of the model was better than random guessing and had predictive value. The top three values of AUC were 0.9351 (PI + MLP), 0.9312 (WRA + MLP), and 0.9306 (PI + AdaBoost). Compared to other models, the performance of MLP model was the best in the weighted acupoint network. Combined with PI indicators, the forecast accuracy was improved significantly. Recall was used to calculate the number of the correct predictions of TP samples. Compared with the accuracy rate, the weighted acupoint network research paid more attention to recall. That is, the fewer prediction errors, the better performance. As shown in Figure 4, the top three values of recall ranking were 0.9209 (WCN + AdaBoost), 0.9085 (WAA + SVM), and 0.8981 (WAA + MLP, PI + MLP). Combining the similarity indices, the performance of AdaBoost, SVM, and MLP was good. The combination of DT with WRA was relatively good. However, the performance of DT combined with other indicators was worse than other models. In particular, the recall value of combination of DT and WPA was the lowest, which reflected the fact that DT model was not suitable in the weighted acupoint network. F1-score was the harmonic average of precision and recall, which was the comprehensive manifestation of the two indicators. As shown in Figure 5, the top three F1-score values were as follows: 0.8757 (PI + MLP), 0.8731 (WRA + SVM), and 0.8713 (WRA + MLP). The combination of WRA index and the four models performed well, which reflected the fact that the stability of WRA index was relatively strong. The experimental results showed that there existed differences in the performance of different similarity indices applied to different models. From the similarity indices, rank of stability was as follows: WRA > WAA > PI > WCN > WPA; predictive performance: PI > WRA > WAA > WCN > WPA. Combining a single similarity index and a fusion similarity index, the prediction performance was not proportional to the number of fusion indices. And there existed a phenomenon that a single index had a negative effect on the fusion index. For example, in a weighted acupoint network, WPA affected the stability of PI. From the perspective of the supervised learning model, MLP, AdaBoost, and SVM showed good adaptability and stability in the weighted acupoint network, especially the combination of MLP and PI, which achieved the maximum value in AUC and F1-score. Combining the performance of similarity indices, PI was selected to combine with four models for the evaluation of performance. As shown in Figure 6, MLP performance was stable and was the best, AdaBoost and SVM were the second, and the indicators of DT were much lower than the other three models.

In summary, in the weighted acupoint network, it is a priority to select PI, WRA, and WAA indicators as similarity indices, and it is a priority to select MLP, AdaBoost, and SVM models as supervised learning models.

## 5. Conclusion

This paper proposes a weighted acupoint network construction method that incorporates the intrinsic and functional properties of acupoints and quantifies the closeness of the links between acupoints through the weight values. The link prediction experiments involved 481 combinations of acupoint combinations, transforming the problem of acupoint combination mining into a problem of the possibility of establishing links between acupoints and confirming the feasibility of applying link prediction to acupoint networks, promoting the development of intelligent acupoint selection for acupuncture treatment of cervical spondylosis and providing a reference for clinical selection. The results of experiment show that the use of weighted network combined with supervised learning has achieved good forecasting performance in the link prediction on the compatibility of acupoints. And the combination of PI + MLP could effectively improve the prediction accuracy. In subsequent studies, we will deepen the network level, enrich the weighting information, and introduce factors that may affect clinical efficacy, such as the direction and depth of needling, in order to broaden the scope of the study and improve the prediction accuracy.

## Figures and Tables

**Figure 1:** Network diagram of weighted acupoints.

**Figure 2:** Experimental flowchart.

**Figure 3:** Forecasting performance of the combination of indicators and models (AUC).

**Figure 4:** Forecasting performance of the combination of indicators and models (recall).

**Figure 5:** Forecasting performance of the combination of indicators and models (F1-score).

**Figure 6:** Forecasting performance based on PI indicators.

**Table 1:** Attributes of acupoints.

Attributes	Number	Elements
Meridian	15	Large intestine meridian (LI), spleen meridian (SP), bladder meridian (BL), pericardium meridian (PC), stomach meridian (ST), conception vessel (CV), small intestine meridian (SI), kidney meridian (KI), lung meridian (LU), gallbladder meridian (GB), triple energizer meridian (TE), heart meridian (HT), liver meridian (LR), governor vessel (GV), extra point

Location	63	Region of oral cavity, toe, ear, knee, back of hand, ankle, sacrum, forearm, head, lateral abdomen, sole, lower abdomen, lateral neck, medial foot, lateral lower leg, medial lower leg, palm, posterior lower leg, anterior wrist, anterior femoral, chest, sternocleidomastoid muscle, inguinal, posterior elbow, umbilical cord, medial hand, anterior forearm, neck, waist, anterior arm, plantar, wrist, posterior arm, lateral thigh, upper lip, upper abdomen, anterior neck, posterior shoulder, forearm, buttocks, triangle muscle, abdomen, face, anterior knee, posterior wrist, palm, anterior shoulder

Indication	670	Contracture pain of leg and foot, pediatric acute wind, acute stomach pain, urinary incontinence, hiccup, elbow numbness, defecation, swelling and pain in the back of hand, lumbosacral pain, fatigue, gall, pain of elbow and arm, blurred vision, axillary swelling, dystocia, upper limb paralysis, arm soreness, pediatric umbilical wind, difficult urination, arm numbness, ulcers, skin itching, shoulder pain, insomnia, fever, palpitation, lower limb paralysis, lack of lactation, hemiplegia, belching, occipital neuralgia, eclipse, pulseless disease, crooked mouth, aphasia, biliary tract ascariasis, sores, addictive rash

## Data Availability

The data included in this paper are available without any restriction upon request to the corresponding author.

## References

[1] Shi X. (2004). *Acupuncture and Moxibustion Therapeutics*.

[2] Zhen Y., Jia-Chun X., Qi-Jing Q., Dao-Yan N., Yu-Liang Z. (2019). Analysis on acupoint selection rules of acupuncture for Alzheimer’s disease based on complex network. *Zhongguo zhen jiu = Chinese acupuncture & moxibustion*.

[3] Wen J., Wang R., Liu J. (2021). Based on complex network analysis of acupuncture and moxibustion treatment of breast hyperplasia, the compatibility of acupoints and the application characteristics of core acupuncture and moxibustion. *Acupuncture Research*.

[4] Jiang L., Yu-Jing H., Tian-Yi Z. (2019). [Rule of acupoint combination in acupuncture treatment of hiccup: a study based on complex network analysis]. *Zhen ci yan jiu = Acupuncture research*.

[5] He Y., Yang F., Yu Y., Grebogi C. (2018). Link prediction investigation of dynamic information flow in epilepsy. *Journal of Healthcare Engineering*.

[6] Turki T., Wei Z. (2017). A link prediction approach to cancer drug sensitivity prediction. *BMC Systems Biology*.

[7] Shen P., Liu S., Wang Y., Han L., Cacace F. (2019). Unsupervised negative link prediction in signed social networks. *Mathematical Problems in Engineering*.

[8] Chen J., Lin X., Jia C. (2019). Generative dynamic link prediction. *Chaos: An Interdisciplinary Journal of Nonlinear Science*.

[9] Ertan B., Mehmet K. (2019). Predicting citation count of scientists as a link prediction problem. *IEEE Transactions on Cybernetics*.

[10] Zhang M., Li P., Xia Y., Wang K., Jin L. (2020). Revisiting Graph Neural Networks for Link Prediction. https://arxiv.org/abs/2010.16103.

[11] Fan H., Zhang F., Wei Y. (2021). Heterogeneous hypergraph variational autoencoder for link prediction. *IEEE Transactions on Software Engineering*.

[12] Niu J., Zhao X., Wu L., Shi X. (2014). Discussing “acupoint sex” again. *Chinese Acupuncture & Moxibustion*.

[13] Zhang Y., Feng Y. (2019). Overview of link prediction methods and development. *Measurement and Control Technology*.

[14] Murata T., Moriyasu S. Link prediction of social networks based on weighted proximity measures.

[15] Lü L., Zhou T. (2010). Link prediction in weighted networks: the role of weak ties. *EPL (Europhysics Letters)*.

[16] Barabasi A., Bonabeau E. (2003). Scale-free networks. *Scientific American*.

[17] An Y., Wang Z., Chen X., Liu L., Li Z., Luo X. (2019). Prediction of latent comorbidity relationship in weighted disease network (Chinese). *Journal of Hunan University*.

[18] Zhao S. (2019). Predicting the links in academic social networks with supervised learning technique (Chinese). *Computer Era*.

